The article "A Novel Fatigue Driving State Recognition and Warning Method Based on EEG and EOG Signals" was published in 2021. Journal: J Healthc Eng.

# A Novel Fatigue Driving State Recognition and Warning Method Based on EEG and EOG Signals

**DOI:** 10.1155/2021/7799793

**Published:** 2021-11-22

**Authors:** Li Liu, Yunfeng Ji, Yun Gao, Zhenyu Ping, Liang Kuang, Tao Li, Wei Xu

**Affiliations:** Jiangsu Vocational College of Information Technology, Wuxi, Jiangsu 214153, China

## Abstract

Traffic accidents are easily caused by tired driving. If the fatigue state of the driver can be identified in time and a corresponding early warning can be provided, then the occurrence of traffic accidents could be avoided to a large extent. At present, the recognition of fatigue driving states is mostly based on recognition accuracy. Fatigue state is currently recognized by combining different features, such as facial expressions, electroencephalogram (EEG) signals, yawning, and the percentage of eyelid closure over the pupil over time (PERCLoS). The combination of these features increases the recognition time and lacks real-time performance. In addition, some features will increase error in the recognition result, such as yawning frequently with the onset of a cold or frequent blinking with dry eyes. On the premise of ensuring the recognition accuracy and improving the realistic feasibility and real-time recognition performance of fatigue driving states, a fast support vector machine (FSVM) algorithm based on EEGs and electrooculograms (EOGs) is proposed to recognize fatigue driving states. First, the collected EEG and EOG modal data are preprocessed. Second, multiple features are extracted from the preprocessed EEGs and EOGs. Finally, FSVM is used to classify and recognize the data features to obtain the recognition result of the fatigue state. Based on the recognition results, this paper designs a fatigue driving early warning system based on Internet of Things (IoT) technology. When the driver shows symptoms of fatigue, the system not only sends a warning signal to the driver but also informs other nearby vehicles using this system through IoT technology and manages the operation background.

## 1. Introduction

Fatigue is a very complex physical and psychological state that can be divided into mental fatigue and physical fatigue. In most cases, mental fatigue and physical fatigue are intertwined and appear at the same time. Mental fatigue is often caused by long-term cognitive activity in the brain. Under brain fatigue, people's cognitive function is limited, and their alertness is reduced. Drivers are prone to both mental and physical fatigue during long-term driving, but mental fatigue is the main problem. Fatigue driving is one of the major hidden dangers of road traffic safety. Research on fatigue driving recognition and early warning technology can reduce the frequency of traffic accidents [1]. Fatigue driving status recognition is a prerequisite for early warning, so fatigue driving status recognition is very important. At present, research on fatigue driving identification methods mainly focuses on three aspects: (1) identification based on driver behavior characteristics: the driver's fatigue state is judged by the recognition of the driver's behavior, such as the movement of the eyelids, the closed state of the eyes [2], and facial expressions [3]. The identification method is simple and easy to implement, but the scoring standard is easily affected by conditions such as personal behavior, light, and image acquisition angle. The collection of various modal data will inevitably be noisy, causing the recognition result to fail to correctly identify the driver's fatigue state. (2) Detection based on vehicle parameters: through the detection of vehicle parameters such as vehicle speed, vehicle position, and steering wheel rotation angle during driving, the driver's operating indicators are obtained, and then the degree of fatigue is judged. Since vehicle parameters are closely related to the actual driving quality of the driver, this method is closer to the actual driving situation. However, vehicle parameters need to be measured during actual operation, which increases the cost of the vehicle. (3) Recognition based on the physiological parameters of the driver: the driver's fatigue state can be judged by identifying the driver's physiological characteristics, such as with electrocardiograms [4], electroencephalograms [5, 6], electrooculograms [7], and electromyography [8, 9].

The article "A Novel Fatigue Driving State Recognition and Warning Method Based on EEG and EOG Signals" was published in 2021. Journal: J Healthc Eng.

Since the EEG signal directly reflects the driver's brain activity and the price of EEG signal acquisition devices are declining, they are therefore convenient to use. Therefore, identifying driving fatigue states based on the EEG signals is considered to be one of the most objective and accurate analysis methods. Reference [5] proposed a new real-time fatigue driving detection method based on EEG signals. The study combines two characteristics of power spectral density (PSD) and sample entropy (SampEn) to judge mental fatigue. The results show that the method is effective for fatigue detection because the prediction results of fatigue are consistent with the phenomena recorded in the simulated driving process. This is considered an objective measure of behavior. Reference [10] proposed a recurrent network-based convolutional neural network (RN-CNN) method to detect fatigue driving. The data used in the experiment are the EEG signals collected during driving simulation. This method can achieve an average recognition accuracy of 92.95%. Reference [11] proposed the detection of the fatigue driving state based on the feature data of sample entropy, approximate entropy, and complexity, which can well identify four different mental fatigue states. Reference [12] uses five different entropies, the relative energy of the alpha wave, and (*θ*+*α*)/*β* as indicators for judging fatigue. The experimental results show that this fusion method can accurately judge the fatigue degree of the driver. Reference [13] uses the fast Fourier transform to extract four rhythm *α*, *θ*, *β*, *δ* features. By analyzing the trend and mutual relationship of these four features, it is found that using (*θ*+*α*)/*β* as the feature to assess the mental state is the most effective. Reference [14] studied sample entropy, fuzzy entropy, approximate entropy, and spectral entropy as the inputs of a decision tree. Experiments have shown that this method has an accuracy of 94% for the identification of fatigue driving, and it can identify fatigue driving more accurately. Typical EEG signal characteristic analysis methods are mainly divided into the time domain [15], frequency domain [16], and time-frequency domain analysis methods [17]. The EEG signal in the frequency domain has obvious characteristics and strong distinguishability. It is of great significance to the analysis of EEG signals. EEG signals in different frequency bands can effectively reflect people's mental state and excitement [18]. Reference [19] uses a convolutional neural network (CNN) to realize emotion recognition based on the time-frequency diagram of EEG signals obtained by a wavelet transform. However, the time-frequency diagram cannot effectively reflect the correlation of EEG signals between different electrodes. The above studies have shown that fatigue driving recognition based on EEGs is the most objective and accurate fatigue recognition method and is known as the “gold standard” of fatigue detection.

The article "A Novel Fatigue Driving State Recognition and Warning Method Based on EEG and EOG Signals" was published in 2021. Journal: J Healthc Eng.

Fatigue driving state recognition based on EOGs mainly separates the horizontal and vertical EOG signals from the electrode signals of the forehead and extracts a series of features, such as gaze, blinking, and saccade, for driver fatigue state recognition. Reference [20] found that as driver fatigue increases, it will be accompanied by long-term blinking, which reflects the relationship between slow eye movement and driver fatigue. By extracting the eye movement features in the EOG signal, machine learning algorithms are used to identify the driver's fatigue state. Reference [21] detected fatigue driving by extracting the fatigue characteristics of blinking, slow eye movement, amplitude, and periodicity in the EOG signal, and the experimental results showed that the detection effect was effective. In summary, driver fatigue detection based on EOG signal characteristics is also feasible.

At present, most studies mainly focus on the fusion of multiple features and the application of integrated classifiers. The purpose of these studies is to maximize the accuracy of fatigue recognition. However, most studies ignore the real-time performance of fatigue driving recognition and early warning. In a real-life environment, the timely identification and early warning of fatigue driving are more meaningful. With the rapid development of modern industry, collection methods of EEG and EOG signals are becoming more advanced. The volume of collection equipment is becoming increasingly miniaturized and portable, their collection accuracy is increasing, and their production cost is decreasing. With the development of Internet of Things (IoT) technology in recent years, it is no longer difficult to collect driver EEG signals without interference. Based on the above background, this paper proposes a fast identification method of fatigue driving based on EEG and EOG. This method can collect the driver's EEG and EOG signals in a real environment and complete rapid identification and timely warning. The contents of this study can be divided as follows:

1. More objective EEG and EOG signal data are used as the identification data of the fatigue driving state. For EEG data, its PSD and differential entropy are extracted as feature data. For EOG, EOG features extracted based on independent component analysis (features_table_ica), EOG features extracted based on subtraction rules (features_table_minus), and EOG features extracted using both subtraction rules and principal component analysis (features_table_icav_minh) are used as feature data. The multifeature data of the two modalities can represent more comprehensive sample information.
2. A fast SVM algorithm based on sample geometric features is proposed. For the case of nonlinear separability, the support vector in the high-dimensional space should also be on the edge of the positive and negative classes. Measured by distance, the support vector is composed of those sample points with larger distances of the same kind and smaller distances of different kinds. The key is to find such sample points. FSVM can greatly reduce the number of training samples and reduce the number of support vectors, resulting in a reduction in the training time of the model, and at the same time, the impact on sample classification accuracy is minimal.
3. Based on the results of fatigue driving status recognition and IoT technology, this paper designs an early warning system. The system can realize data collection, identification, and early warning. When a driver is detected to be fatigued, the system not only sends a warning signal to the driver but also informs other nearby vehicles using this system through the Internet of Things technology and manages the operation background.

The article "A Novel Fatigue Driving State Recognition and Warning Method Based on EEG and EOG Signals" was published in 2021. Journal: J Healthc Eng.

## 2. Related Information

### 2.1. EEG Multifeature Extraction Method

#### 2.1.1. Differential Entropy Feature Extraction

The differential entropy feature is expanded on the basis of Shannon entropy. In 2013, differential entropy was used for the first time to characterize EEG characteristics. Compared with the traditional PSD, it shows superior performance [22]. The original definition of calculating differential entropy is as follows:

(1) $$\begin{array}{c} h\left(x_{n}\right)=-\int_{X}f\left(x\right)\log\left(f\left(x\right)\right)\text{d}x. \end{array}$$

When a random variable follows the Gaussian distribution *N*(*u*, *σ*^2^), the differential entropy can be simply calculated by the following formula:

(2) $$\begin{array}{c} h\left(X\right)=-\int_{-\infty }^{+\infty }f\left(x\right)\log\left(f\left(x\right)\right)\text{d}x=\frac{1}{2}\log\;2\pi e\sigma^{2}, \end{array}$$

where $f\left(x\right)=1/\sqrt{2\pi \sigma^{2}}\exp{\left(x-\mu \right)}^{2}/2\sigma^{2}$.

#### 2.1.2. PSD Feature Extraction

PSD is used to characterize the change in signal power with changes in frequency. In practical applications, the average value of the signal value in a certain frequency band is generally regarded as the PSD of the frequency band, and the calculation formula is

(3) $$\begin{array}{c} p\left(x_{n}\right)=\frac{1}{N}X\left(x_{n}\right)X^{*}\left(x_{n}\right), \end{array}$$

where *X*(*x*_*n*_) is the discrete Fourier change value of segment *n* and *X*^*∗*^(*x*_*n*_) is the conjugate function of *X*(*x*_*n*_).

### 2.2. Typical Classification Model

Table 1 gives the relevant introduction of each commonly used classification model. At present, the classification model of fatigue driving state recognition can be divided into machine learning [23, 24] and deep learning [25, 26]. The mathematical model of the machine learning algorithm is simple, and the algorithm time complexity is relatively low, but the recognition accuracy is not as good as that of the deep learning algorithm. The model of the deep learning algorithm is complex, there are many parameters that need to be adjusted, and the time complexity of the algorithm is high, but the recognition rate of the algorithm is high. In summary, the two types of classification models have their own characteristics and applicable scenarios. Since the scenarios used in this article do not belong to the category of large samples and fatigue driving recognition and early warning have high real-time requirements, the machine learning algorithm can fully meet the requirements. Therefore, the classic SVM in machine learning is used as the basic algorithm to classify datasets.

The article "A Novel Fatigue Driving State Recognition and Warning Method Based on EEG and EOG Signals" was published in 2021. Journal: J Healthc Eng.

### 2.3. Labeling of Fatigue Signal Labels

The key to fatigue identification based on EOG is calculating the PERCLOS value. The PERCLOS value indicates the degree of closure of the eyelids per unit time. The calculation formula is as follows:

(4) $$\begin{array}{c} \text{PERCLOS}=\frac{\text{eye}\_\text{closing}\_\text{time}}{\text{total}\_\text{time}}. \end{array}$$

PERCLOS is marked as *P*, and the threshold of *P* is set to determine whether it is fatigued. When *P* < 0.35, it indicates that the driver is awake. When *P* > 0.35, it indicates that the driver is tired. According to different *P* values, two different states can be obtained. This type of research can be described as a binary classification task. The awake state is recorded as 0, and the fatigue state is recorded as 1.  Table 2 shows the specific labeling method.

### 2.4. ZigBee Wireless Technology

The ZigBee standard is a wireless ad hoc network standard suitable for wireless sensor networks proposed by the ZigBee Alliance in 2004. ZigBee chips usually integrate basebands, microcontrollers, and memory, and ZigBee can work in the frequency bands of 868 MHz, 915 MHz, and 2.4. The data transmission rate of the ZigBee network ranges from 20 to 900 kpbs. Each ZigBee network contains a coordinator, and the task of the coordinator allows the router to expand the communication range of the network. Since ZigBee nodes can wake up from sleep in 30 ms, which makes ZigBee's response delay far lower than other types of wireless technologies, ZigBee is very suitable for small data volume burst data transmission. The system designed in this paper will not only alert drivers of fatigue but also transmit alerts to other vehicles. This requires the establishment of a suitable wireless network connection between the vehicles. Since the driver is not always in a state of fatigue, the exchange of data between vehicles will be intermittent, and there will be no continuous data exchange. Moreover, the amount of data carried by each fatigue alert is very small. Based on the above analysis, this article selects a ZigBee network suitable for sudden small data transmission. As a typical protocol for wireless sensor networks, ZigBee is suitable for the transmission of such data. Therefore, this article selects ZigBee as the wireless network standard between vehicles.

## 3. Fatigue Driving Status Recognition and Early Warning System

### 3.1. System Framework

In this study, a rapid fatigue state recognition and early warning system was designed. The architecture of the system is shown in Figure 1. The hardware system of the whole system mainly includes a Bluetooth headset and a vehicle-mounted terminal. The Bluetooth headset is mainly responsible for collecting EEG and EOG signals. Through the Bluetooth communication protocol, the data are transmitted to the vehicle terminal for storage, processing, and analysis. The fatigue state recognition module in the vehicle terminal is responsible for classifying the received EEG and EOG signals to determine whether the driver is tired. When the result of the identification is fatigue, a warning message will be issued to the driver, operation manager, and surrounding vehicles. A set of equipment can be installed on each vehicle, and the system includes a sending end and a receiving end.

The article "A Novel Fatigue Driving State Recognition and Warning Method Based on EEG and EOG Signals" was published in 2021. Journal: J Healthc Eng.

### 3.2. Recognition Model

This study uses a fast SVM model to classify feature data. For nonlinearly separable data, the support vector in the high-dimensional space should also be on the edge of the positive and negative classes. Measured by distance, the support vector is composed of those sample points with a larger distance from the same class and a smaller distance from the heterogeneous group. The key is to find such sample points. First, the distance between any two points is described. The following mapping formula is used:

(5) $$\begin{array}{c} \phi :x\in R^{P}⟶\phi \left(x\right)\in R^{m},m>p,\;\forall x_{i},x_{j},x_{j}\in R^{P}. \end{array}$$

The distance between any two points is defined in space *R*^*m*^:

(6) $$\begin{array}{c} d\left(\phi \left(x_{i}\right),\phi \left(x_{j}\right)\right)=\left\|\phi \left(x_{i}\right)-\phi \left(x_{j}\right)\right\|,\\ =\sqrt{\left(\phi \left(x_{i}\right)-\phi \left(x_{j}\right)\right)\cdot \left(\phi \left(x_{i}\right)-\phi \left(x_{j}\right)\right)}\\ =\sqrt{\phi \left(x_{i}\right)\cdot \phi \left(x_{i}\right)-2\phi \left(x_{i}\right)\cdot \phi \left(x_{j}\right)+\phi \left(x_{j}\right)\cdot \phi \left(x_{j}\right)}\\ =\sqrt{K\left(x_{i},x_{i}\right)-2K\left(x_{i},x_{j}\right)+K\left(x_{j},x_{j}\right)}\\ =\sqrt{2-2K\left(x_{i},x_{j}\right)}. \end{array}$$

Assume sample point *z*_*k*_ ∈ *G*^+^; for any *k* ∈ *I*^+^, it corresponds to point *ϕ*(*z*_*k*_) in the high-dimensional space.

A pair of distance values (*d*_*k*_^+^, *d*_*k*_^−^) is assigned to point *ϕ*(*z*_*k*_),

(7) $$\begin{array}{c} \left\{\begin{array}{c} d_{k}^{+}=\frac{1}{l^{+}}\sum_{i\in I^{+}}d\left(\phi \left(z_{k}\right),\phi \left(x_{i}\right)\right),\\ d_{k}^{-}=\frac{1}{l^{-}}\sum_{i\in I^{+}}d\left(\phi \left(z_{k}\right),\phi \left(x_{j}\right)\right). \end{array}\right. \end{array}$$

The parameter *r* represents the proportion of possible support vectors in the training sample set. There are critical values c1 and c2 such that *P*{*d*_*k*_^+^ > *c*_1_}=*r* and *P*{*d*_*k*_^−^ < *c*_2_}=*r*. That is, we find those points *ϕ*(*z*_*k*_) with a larger average distance from the positive point and a smaller average distance from the negative point. The support vector is the point *z*_*k*_ that satisfies the condition {*ϕ*(*z*_*k*_)*|d*_*k*_^+^ > *c*_1_, *d*_*k*_^−^ < *c*_2_, *k* ∈ *I*^+^}. As shown in Figure 2, the points in set *T*_1_^+^={*ϕ*(*z*_*k*_)*|d*_*k*_^+^ > *c*_1_, *k* ∈ *I*^+^} correspond to the points in the shape of ① in the figure. The point in *T*_2_^+^={*ϕ*(*z*_*k*_)*|d*_*k*_^−^ < *c*_2_, *k* ∈ *I*^+^} corresponds to point ② in the figure. Then, point *ϕ*(*z*_*k*_) ∈ *T*^+^,*T*_1_^+^∩*T*_2_^+^. In the same way, for *z*_*k*_ ∈ *G*^−^ and any *k* ∈ *I*^−^, set *T*^−^ can be found. Then, the set formed by the support vector is *T*^*B*  *D*^=*T*^+^ ∪ *T*^−^.

The article "A Novel Fatigue Driving State Recognition and Warning Method Based on EEG and EOG Signals" was published in 2021. Journal: J Healthc Eng.

The FSVM algorithm follows a certain principle of the distance between samples to extract support vectors, which are used as training samples for the SVM, and then the SVM is used for training. The implementation steps of the algorithm are 5 in total, and details of each step are shown below:

**Step 1 .**

Set the scale parameter *r*(0 < *r* < 1).

**Step 2 .**

In the high-dimensional space, calculate the distance matrix $D={\left(d_{ij}\right)}_{l\times l}\left[\begin{array}{cc} D_{11} & D_{12}\\ D_{21} & D_{22} \end{array}\right]$, where $d_{ij}=d\left(\phi \left(x_{i}\right),\phi \left(x_{j}\right)\right)=\sqrt{2-2K\left(x_{i},x_{j}\right)}$. *D*_11_(*D*_22_) represents the block matrix formed by the distance between any two points in the positive and negative sets. *D*_12_(*D*_21_) represents the block matrix formed by the distance between each point of the positive and negative clusters.

**Step 3 .**

Calculate the average matrix $V={\left[\begin{array}{cc} V_{11} & V_{12}\\ V_{21} & V_{22} \end{array}\right]}_{\left(l^{+}+l^{-}\right)\times 2}$. Set *I*_*l*^+^_=1/*l*^+^*e*_*l*^+^×1_, *I*_*l*^−^_=1/*l*^−^*e*_*l*^−^×1_; then *V*_11_=*D*_11_*I*_*l*^+^_, *V*_12_=*D*_12_*I*_*l*^−^_, *V*_21_=*D*_21_*I*_*l*^+^_, and *V*_22_=*D*_22_*I*_*l*^−^_.

**Step 4 .**

Extract the support vector set according to the given ratio *r*. Sort the components in *V*_11_ and *V*_22_ in descending order. Sort the components in *V*_12_ and *V*_21_ in ascending order. Extract the top *l*^+^ · *r* and *l*^−^ · *r* samples after sorting to form a new training set *T*^*B*  *D*^(|*T*^*B*  *D*^| < *l* · *r*).

The article "A Novel Fatigue Driving State Recognition and Warning Method Based on EEG and EOG Signals" was published in 2021. Journal: J Healthc Eng.

**Step 5 .**

The SVM algorithm is trained on *T*^*BD*^ to obtain the final model.

## 4. Experiment

### 4.1. Introduction to Simulation Data

The SEED-VIG [27] dataset was used for experimental simulation, which is mainly composed of EEG and EOG signals. To collect the dataset in the real scene, the data collector used the Neuroscan system to collect the relevant signals of the driver in the simulated driving environment. The sampling frequency is 1 kHz, and 21 channels of data are collected in total. The electrode position during EOG acquisition is shown in Figure 3(a), and there are 4 channel electrodes in total. The electrodes set for the EEG signal are 6 channels in the temporal brain area and 11 channels in the back brain area. The specific electrode positions are shown in Figure 3(b). The placement of these positions meets the international 10–20 electrode distribution requirements.

The collected initial EEG signal contains problems such as noise, which requires preprocessing, feature extraction, and smoothing operations on signals from different brain regions. The different brain areas mainly include the temporal lobe brain area, *T* area; the occipital brain area, *P* area; the prefrontal EEG, F area; and the brain area signal leads, bandwidth, and characteristic dimensions, which are shown in Table 3. First, the forehead EEG is separated from the forehead electrode signals, and the EEG signals of each brain area are divided into 5-band EEG signals. The features of EEG and EOG data are extracted, as shown in Table 4.

### 4.2. Experimental Setup

During the experiment, the main contrastive algorithms used are BP [28], RF [29], SVM [30], and CNN [31]. Both SVM and FSVM use a radial basis kernel function, and the kernel function parameter is set to 0.001. The parameters of the other comparison algorithms are the same as those in the reference. The evaluation index of the model used is the recognition accuracy rate, and its calculation formula is as follows:

(8) $$\begin{array}{c} \text{Acc}=\frac{TP+TN}{TP+TN+FP+FN}. \end{array}$$

The computer configuration information used in the experiment is 32 G of memory, an i7-11700F CPU, a Win10 operating system, and the MATLAB 2020a programming tool.

### 4.3. Experimental Results and Analysis

#### 4.3.1. Fatigue Recognition Accuracy Rate Experiment

The dataset is randomly divided into a training set and a test set at a ratio of 7 : 3. First, the EEG feature and EOG feature are classified separately using the classifier and then the two features are combined for classification. The experimental data are the mean value after running the algorithm 10 times. The experimental results are shown in Tables 5–7.

The article "A Novel Fatigue Driving State Recognition and Warning Method Based on EEG and EOG Signals" was published in 2021. Journal: J Healthc Eng.

The data in Table 5 show that, for most classification algorithms, the recognition rate based on DE features is slightly better than that based on PSD features. This shows that the evaluation effect based on the DE feature is better than that based on the PSD feature. Regarding the recognition accuracy index, regardless of whether it is based on PSD or DE features, the recognition rate of the CNN deep learning algorithm is significantly ahead of that of the machine learning algorithm. This shows that, in terms of recognition accuracy, the performance of deep learning algorithms is significantly better than that of machine learning algorithms. Among the machine learning algorithms, the SVM algorithm has the best recognition rate. This is also the reason why SVM is chosen as the basic algorithm. The recognition accuracy of FSVM is comparable to that of classic SVM.

The data in Table 6 show that, for different classification algorithms, the recognition rate based on the features_table_icav_minh feature is the best. This shows that the classification information carried by the EOG features extracted by both subtraction rules and principal component analysis is more abundant. Among the different classification algorithms, CNN has the highest recognition rate, which shows that the recognition effect of deep learning algorithms is indeed very good. The recognition rates of SVM and FSVM are similar, and the recognition rate of FSVM is slightly higher.

To explore the influence of multimodal data on the recognition accuracy, EEG and EOG signals were fused for experimental analysis. EEG uses differential entropy feature data, using the average of the three brain regions P, *T*, and F as the final experimental data. EOG uses the features_table_icav_minh feature with the best recognition effect as the input feature data. The recognition results of the fusion features of each algorithm are shown in Table 7.

The experimental data shown in Table 7 show that, in addition to the BP algorithm, the recognition accuracy of other algorithms based on fusion features is better than the recognition accuracy of a single feature. This shows that the fusion feature can effectively improve the fatigue recognition accuracy. The changes in the recognition accuracy of each algorithm based on different features are shown in Figure 4. It can be clearly seen from the figure that the recognition rate of CNN and FSVM based on fusion features has the largest increase, followed by SVM, and RF has the smallest increase. The recognition accuracy of the BP algorithm has declined to a certain extent. In summary, the use of fusion features has advantages in the recognition rate.

The article "A Novel Fatigue Driving State Recognition and Warning Method Based on EEG and EOG Signals" was published in 2021. Journal: J Healthc Eng.

#### 4.3.2. Fatigue Recognition Model Training Time Consumption Experiment

The recognition model is trained based on the fusion features, and the time taken to train the model 10 times is averaged. The training time consumption details of each model are shown in Table 8. The data in Table 8 show that the time spent on machine learning algorithms is lower than the time spent on deep learning algorithms. For scenarios that require a quick response time, machine learning algorithms are more suitable. Among the many machine learning algorithms, the training time required for the FSVM model mentioned in this article is greatly reduced. Compared with the classic SVM model, the training time is reduced by 33.95%. Compared with the CNN, the training time of the FSVM model is only a quarter of it. In summary, the model proposed in this paper can not only ensure a better recognition rate but also reduce the training time for the model. Therefore, it can fully meet the task of real-time fatigue identification and has good practical value.

## 5. Conclusion

The rapid identification and early warning of the fatigue driving state are the key to reducing traffic accidents. Quick and accurate fatigue identification is a prerequisite for effective early warning. This study is based on two-modal data of EEGs and EOGs to identify the fatigue driving state and extracts multiple features of the two-modal data for experimental analysis. Experimental data show that the fatigue state recognition accuracy of multimodal data fusion is higher. In the selection of classification models, deep learning algorithms have a leading advantage, and the recognition accuracy is higher than that of machine learning algorithms. However, considering the real-time requirements of fatigue state recognition tasks, this study proposes an FSVM algorithm that can quickly provide model training. The FSVM algorithm greatly improves the training speed of the model without reducing the recognition accuracy and achieves the expected effect. On the other hand, based on fast and accurate recognition results, this article designed a set of early warning systems based on IoT technology to extend the early warning information from a single vehicle to the Internet of Vehicles. When the driver is in a fatigue state, the system can not only send a warning signal to the driver but also notify other nearby vehicles using this system and manage the operation background through IoT technology. Regarding the identification of fatigue status, the next step of this research will be to improve the accuracy of identification, and more modal data can be introduced for comprehensive decision-making. In an early warning system, when the vehicle speed is too high and the distance is too large, the signal between the vehicle and other vehicles is likely to be weak, and it is impossible to guarantee the successful warning of other vehicles. LoRa has the characteristics of long communication distance, low power consumption, and low cost, which may be able to solve the above problems. This is also the content of this study, which needs further research in the future.

The article "A Novel Fatigue Driving State Recognition and Warning Method Based on EEG and EOG Signals" was published in 2021. Journal: J Healthc Eng.

## Figures and Tables

**Figure 1:** System structure diagram.

**Figure 2:** Distribution of sample points based on distance analysis.

**Figure 3:** Electrode position during EOG and EEG acquisition.

**Figure 4:** Recognition accuracy of each algorithm based on different features.

**Table 1:** Typical classification model.

Model	Main idea	Advantages and disadvantages
Artificial neural network (ANN)	There are three types of processing units in the network: input unit, output unit, and hidden unit. The input unit receives signals and data from the outside world. The output unit realizes the output of system processing results. A hidden unit is a unit that lies between an input and output unit and cannot be viewed from outside the system. ANN is a kind of nonprogrammed, adaptive, and brain-style information processing mode, whose essence is to obtain a parallel and distributed information processing function through network transformation and dynamic behavior.	Advantages: ① it is a simple application; ② it has more accurate classification results; and ③ it has the ability to quickly search for optimization. Disadvantages: ① it easily enters the local optimum.

SVM	The algorithm finds a dividing hyperplane that can correctly separate the two types of data on both sides to achieve the effect of data classification and prediction. This hyperplane is determined by the support vectors.	Advantages: ① the “curse of dimensionality” can be avoided; ② it has a known effective algorithm that can be used to find the global minimum of the objective function; ③ the generalization ability of the algorithm is good. Disadvantages: ① it is difficult to implement large-scale training samples; ② it has difficulty solving the multicategory problem; ③ it is sensitive to parameter and kernel function selection.

Random Forest (RF)	The forest is composed of many trees, so the result of RF depends on the decision result of multiple trees. This is an integrated learning idea. For example, there is a new animal in the forest, and the forest holds a forest meeting to determine what kind of animal it is. Every tree must express its opinions. The result with the most votes will be the final result.	Advantages: ① it can handle very high-dimensional (many features) data, and there is no need to perform feature selection; ② the training speed is fast, and it is easy to make a parallel method; ③ the implementation is relatively simple. Disadvantages: ① it is prone to overfitting; ② for data with attributes with different values, the attribute weights produced by RF on such data are unreliable.

AdaBoost	The algorithm trains several individual learners with a certain combination strategy so that a strong learner can finally be formed to achieve the goal of more people and more power.	Advantage: ① under the framework of AdaBoost, various classification models can be used to build weak learners, which is very flexible; ② given its high precision, it can be applied to most classifiers without the need to adjust parameters. Disadvantages: ① unbalanced data leads to a decrease in classification accuracy; ② training is time-consuming.

CNN	A method consisting of the following layered form: input layer: data entry Convolutional layer: for feature extraction Pooling layer: used to extract features again Hidden layer: the layer in the middle Fully connected layer: after vectorizing the extracted feature matrix, classify its features.	Advantages: it has a high classification accuracy rate. Disadvantages: ① parameters need to be adjusted; ② it needs large amount of data; ③ it requires a large amount of calculation.

The article "A Novel Fatigue Driving State Recognition and Warning Method Based on EEG and EOG Signals" was published in 2021. Journal: J Healthc Eng.

**Table 2:** Fatigue marking status.

*P* value range	State	Label
*P* < 0.35	Wide awake	0
*P* > 0.35	Fatigue	1

**Table 3:** Signal distribution and characteristic dimensions of brain regions.

Brain area	Signal lead	Characteristic frequency band	Feature dimension
P	11	*δ*, *θ*, *α*, *β*, *γ*	55
T	6	*δ*, *θ*, *α*, *β*, *γ*	30
F	4	*δ*, *θ*, *α*, *β*, *γ*	20

**Table 4:** EEG and EOG characteristics.

Signal	Feature extraction method	Feature
EEG	Short-time Fourier transform	Power spectral density linear dynamic system smoothing characteristics (PSD).
		Smoothing characteristics of differential entropy linear dynamic system (DE).

EOG	Wavelet transform peak detection method	Electroocular features extracted based on independent component analysis (features_table_ica). Eye electrical features extracted based on subtraction rules (features_table_minus). Electrooculogram features extracted by fusion of subtraction rules and principal component analysis (features_table_icav_minh).

**Table 5:** Recognition accuracy based on EEG features.

Brain area	Feature	BP	RF	SVM	CNN	FSVM
P	PSD	0.8892	0.8791	0.9146	0.9287	0.9128
	DE	0.8957	0.8880	0.9245	0.9420	0.9215

T	PSD	0.8921	0.8687	0.9112	0.9117	0.9126
	DE	0.8985	0.8763	0.9197	0.9421	0.9204

F	PSD	0.8864	0.8725	0.9020	0.9223	0.9043
	DE	0.8903	0.8804	0.9189	0.9468	0.9180

Mean	PSD	0.8892	0.8734	0.9093	0.9209	0.9099
	DE	0.8948	0.8816	0.9210	0.9436	0.9200

The article "A Novel Fatigue Driving State Recognition and Warning Method Based on EEG and EOG Signals" was published in 2021. Journal: J Healthc Eng.

**Table 6:** Recognition accuracy based on EOG features.

Algorithm	features_table_ica	features_table_minus	features_table_icav_minh
BP	0.9032	0.9104	0.9131
RF	0.9153	0.9086	0.9178
SVM	0.9343	0.9357	0.9406
CNN	0.9481	0.9396	0.9484
FSVM	0.9391	0.9325	0.9412

**Table 7:** Recognition accuracy rate of fusion features.

Algorithm	EEG	EOG	EEG + EOG
BP	0.8948	0.9131	0.9124
RF	0.8816	0.9178	0.9209
SVM	0.9210	0.9406	0.9478
CNN	0.9436	0.9484	0.9517
FSVM	0.9200	0.9412	0.9511

**Table 8:** Training time.

Model	BP	RF	SVM	CNN	FSVM
Time (s)	286	225	217	639	162

## Data Availability

The labeled dataset used to support the findings of this study is available from the corresponding author upon request.
